The article "Methyltransferase-like 14 silencing relieves the development of atherosclerosis via m6A modification of p65 mRNA" was retracted in 2026. Reasons: plagiarized images; overlap with other authors' work; original data or images not available; concerns about the data.

# Methyltransferase-like 14 silencing relieves the development of atherosclerosis via m^6^A modification of p65 mRNA

**DOI:** 10.1080/21655979.2022.2031409

**Published:** 2022-05-11

**Authors:** Yingjie Liu, Gang Luo, Quan Tang, Yang Song, Daxing Liu, Hongjuan Wang, Junliang Ma

**Affiliations:** a Department of Cardiac and Vascular Surgery, Affiliated Hospital of Zunyi Medical University, Zunyi, China; b Department of Scientific Research, Affiliated Hospital of Zunyi Medical University, Zunyi, China; c Department of Thoracic Surgery, Affiliated Hospital of Zunyi Medical University, Zunyi, China

**Keywords:** METTL14, atherosclerosis, aorta, m^6^A, p65

## Abstract

To explore the METTL14-dependent m^6^A modification mechanism involved in the development of atherosclerosis. Oxidized low-density lipoprotein (ox-LDL) and the HUVEC cell line were used to establish an atherosclerosis cell model in vitro, and *APOE*^−/−^ mice fed a high-fat diet were used as the animal model. Cell viability and apoptosis were assessed using MTT assays and flow cytometry. The status of m^6^A in HUVECs was examined using MeRIP-qPCR. Oil Red O staining was used to evaluate the lesions or plaques on aortas separated from the target mice. METTL14 and METTL3 were upregulated in HUVECs after ox-LDL treatment. After transfection with si-METTL14, the bcl-2 expression level and the viability of ox-LDL-incubated cells increased, whereas the apoptosis rate and the expressions of Bax and cleaved caspase-3 decreased. However, the effect of METTL14 knockdown was reversed by p65 overexpression. After METTL14 knockdown, there was a decrease in the total m^6^A content in HUVECs, m^6^A modification, and p65 expression. The plaques and lesion areas on the high-fat diet *APOE***^−/−^** mouse aortas were smaller after METTL14 silencing. METTL14 reduced cell viability and promoted apoptosis of HUVECs, which were both induced by ox-LDL via m^6^A modification of p65. Knocking down METTL14 could inhibit the development of atherosclerosis in high-fat diet-treated *APOE***^−/−^** mice.

## Highlight

- METTL14 expression was upregulated in AS
- The p65 mRNA was a potential m6A target for METTL14
- Overexpressing p65 reversed the si-METTL14 effects

## 1. Introduction

The development of the social economy and changes in people’s lifestyles have led to high incidence and mortality rates for coronary heart disease [1]. Its mortality rate exceeds that of tumors and other diseases, and ranks first as a cause of death [2]. It has become a major public health problem and exploring effective methods to prevent coronary heart disease is a top priority. Atherosclerosis (AS) is the main pathological basis of coronary heart disease and impaired endothelial function is an early key event in the mechanism controlling AS [3]. The deposition of oxidized low-density lipoprotein (ox-LDL) in the subendothelial layer of blood vessels is the main cause of AS [3]. Studies have shown that ox-LDL can cause vascular endothelial cell damage, leading to the infiltration of lipid components and inflammatory cells into the damaged area and the gradual formation of atheromatous plaques [4]. Therefore, inhibition of ox-LDL-induced vascular endothelial cell damage is particularly important for the prevention and treatment of AS.

Methylation of m^6^A RNA is mainly regulated by methyltransferase-like 3 (METTL3), methyltransferase-like 14 (METTL14), and Wilms tumor 1-associated protein (Wilms tumor 1-associated protein, WTAP) [5]. The m^6^A modification is one of the most abundant methylation modifications to RNA and has become an important research area in recent years. The modification mainly consists of the transferal of methyl groups catalyzed by methylase, demethylase and uses binding proteins that are able to recognize specific-binding sites [6]. The modification of m^6^A (N6-methyladenosine) plays an important role in the function of RNA and is related to the pathological process of many diseases, especially cardiovascular diseases [7]. The m^6^A methylation process mainly affects vascular endothelial cells, macrophages, and vascular smooth muscle cells, and its methylation in these cells leads to the occurrence and development of AS [8]. Quiles-Jiménez et al. [9] used mass spectrometry to analyze the m^6^A levels in non-atherosclerotic arteries and carotid atherosclerotic tissues and found that m^6^A methylase and demethylase levels in atherosclerotic tissues had changed.

The aim of this study was to explore the mechanism underlying METTL14-dependent m^6^A modification during the development of AS. We hypothesized that METTL14 significantly increased during the injury period, but METTL14 knockdown significantly inhibited AS progression. Mechanistically, METTL14 specifically targets p65 mRNA to regulate m^6^A modification and the stability of p65 mRNA.

## 2. Methods and materials

### 2.1. Animal model

Thirty 8-week old male *APOE*^−/−^ C57BL/6 J mice were purchased from Beijing Vital River Laboratory Animal Technology Co., Ltd., China. All procedures associated with the animal experiments were performed according to the 3 R principle and approved by the Zunyi Medical University Animal Ethics Committee. The mice were randomly divided into control, Ad-sh-NC, and Ad-sh-METTL14 groups (10 mice per group). The mice in the control group were fed a normal diet, while the Ad-sh-NC and Ad-sh-METTL14 groups were fed a high-fat diet (20% fat and 0.25% cholesterol). Furthermore, 300 μL of constructed sh-NC or sh-METTL14 adenovirus was injected every 3 weeks into the caudal veins of mice from the Ad-sh-NC or Ad-sh-METTL14 groups, respectively. The constructed vectors were obtained from HanBio Technology Co., Ltd. (Shanghai, China). All mice were sacrificed after 24 weeks and the aortas were separated for further experiments.

### 2.2. Cell culture and transfection

Human umbilical vein endothelial cell line (HUVECs, EAhY926) purchased from the ATCC was used in the experiment. The cells were cultured with DMEM medium supplemented with FBS (10%). 100 μL/mL of ox-LDL was added in the medium and incubated with target cells for 12 h or 24 h to establish cell models for atherosclerosis. si-NC and si-METTL14 purchased from GenePharma (Shanghai, China) were transfected into HUVECs by Lipofectamine 2000 (Invitrogen, CA, USA). pcDNA 3.1-p65 or pcDNA 3.1-NC adenoviral vectors obtained from HanBio Technology Co. Ltd. (Shanghai, China) were transfected into HUVECs for the overexpression of p65 or used as a control in the following experiment.

### 2.3. MTT assays

As described by Präbst et al. [10], the cells were cultured in 96-well plates at a density of 2 × 10^3^/mL. After treatment, the cells were incubated with 10 μL MTT solution (0.5 mg/mL; Beyotime, Shanghai, China) for 4 h. A spectrophotometer (BioTek, Winooski, VT, USA) was used to measure absorbance at 490 nm. The absorbance represents cell viability.

### 2.4. Flow cytometry

An Annexin V PE/7-AAD tool kit (Solarbio, Beijing, China) was used to detect apoptosis according to a previous study [11]. The cells were first resuspended at a density of 1 × 10^5^/mL and then added to the flow tubes. The cells were detected using a flow cytometer (BD, Franklin Lakes, NJ, USA) after incubation with Annexin V PE and 7-AAD, according to the manufacturer’s protocol. The apoptosis rates were analyzed by ModFit LT software.

### 2.5. Western blot

As described by Taylor et al. [12], the total protein was first collected from cells with a RIPA lysis buffer (Solarbio) and then quantified with a BCA protein assay kit (Solarbio). After electrophoresed on SDS-PAGE, the samples were then transferred onto PVDF membranes (Millipore, MA, USA) and blocked with 5% nonfat milk for 1 h at room temperature. The primary antibody of Anti-Bax (Abcam, Cambridge, UK), Anti-Cleaved Caspase-3 (Abcam, Cambridge, UK), Anti-Bcl-2 (Abcam, Cambridge, UK), Anti-NF-kB p65 (Abcam, Cambridge, UK) and the secondary antibodies of HRP conjugated Goat-anti-Rabbit IgG (1:10,000, Invitrogen) were used for the incubation. After reacting with ECL reagent (Millipore, MA, USA), the samples were then examined in a Bio-Rad imaging system (Hercules, CA, USA). Image J software was used to measure the gray value of each sample.

### 2.6. Determination of the cholesterol, triglyceride, LDL-cholesterol, and HDL-cholesterol levels

The cholesterol, triglyceride, LDL-cholesterol, and HDL-cholesterol levels in the blood of the mice were determined with corresponding kit provided by Nanjing Jiangcheng Bioengineering Institute (Nanjing, China). All operations shall be carried out in strict accordance with the requirements of the kits.

### 2.7. Oil Red O staining

The Oil Red O staining was performed as a previous study [13]. After fixing with 4% paraformaldehyde and washing with PBS, the aortas were treated with Oil Red O (Solarbio), which had been dissolved in isopropyl alcohol for 1 h. The samples were washed with 60% isopropanol and water and then photographed. The tissue separated from the aortic root was dehydrated with 15% and 30% sucrose and embedded in optimal cutting temperature compound. The samples were then frozen in liquid nitrogen and cut into 8 μM slices for Oil Red O (Solarbio) staining. The plaque area of the aortas and the lesion area of the aorta root were analyzed using Image J software.

### 2.8. TUNEL staining

According to a previous study [14], TUNEL staining was carried out according to the instructions of Dead EndTM Fluorometric TUNEL System Kit (Promega company, USA). The specific steps are as follows: the tissue was deparaffinized and digested with proteinase K (20 μg/ml). After washing with PBS, the sections were mixed with 100 μl Equilibration Buffer and TUNEL reaction mixture and incubated at 37°C in the dark for 60 min. After that, DAPI was added. Finally, the sections were washed with PBS and mounted with glycerol. A fluorescence microscope was used to observe the sections.

### 2.9. Immunofluorescence

According to a previous study [15], the tissue sections were fixed with 4% paraformaldehyde, and then the goat serum working solution, primary antibody, secondary antibody, and DAPI were added in sequence to incubate on the tissue, in which the dilution of CD31 antibody was 1 : 200 (BD Pharmingen, USA). Finally, the sections were observed under the fluorescent microscope,

### 2.10. RT-qPCR assay

Trizol reagent (Invitrogen) was used to extract the total RNA. A GoScript™ Reverse Transcription System (Promega, WI, USA) was used for the synthesis of cDNAs. Then, an SYBR Premix EX Taq (Takara, Dalian, China) was used to treat the samples. Real-time PCR reaction was performed in a CFX96 Real-Time PCR Detection System (Bio-Rad, Hercules, CA, USA). The primers were purchased from Sangon Biological Engineering Technology company (Shanghai, China). The 2^−ΔΔCt^ [16] was calculated for the calculation.

### 2.11. RNA m^6^A quantification and MeRIP-qPCR

An m^6^A RNA Methylation Assay Kit (Abcam, Cambridge, UK) was used to examine the m^6^A content [17]. Extracted RNA (150 ng) and the relevant solution were added to a 96-well plate according to the manufacturer’s protocol. The absorption was detected using a microplate reader at 450 nm, and the percentage m^6^A content was calculated. A Dynabeads™ mRNA Purification Kit (Invitrogen, Waltham, MA, USA) was used in the MeRIP-qPCR assay to isolate the mRNA from the extracted total RNA [18]. One-third of the isolated samples were used as an input control. The primary anti-N6-methyladenosine (Abcam) or rabbit IgG (Abcam) antibody was incubated with Pierce™ Protein A/G Magnetic Beads (Thermo Scientific, Waltham, MA, USA) for conjugation. It was then mixed with the rest of the isolated samples for precipitation with the aid of glycogen, sodium acetate, and ethanol. Any m^6^A enrichment was evaluated by qPCR and calculated by normalizing the results to the input.

### 2.12. ROS detection

2’,7’-dichlorofluorescin diacetate (DCFH) (Sigma, USA) was applied to detect the level of ROS. Briefly, at the indicated harvest time point, the cells were rinsed with PBS (4°C). Then, the cells were incubated with DCFH (10 μM) at 37°C for 30 min in a dark setting. The fluorescence intensity of harvested cells were detected with Flow Cytometry. The acquired data were analyzed by Flowjo_V10.

### 2.13. Enzyme linked immunosorbent assay (ELISA)

The cell culture supernatant was taken and centrifuged in a 4°C centrifuge (2000 r/min, 5 min), and the supernatant was collected and stored at −80°C for testing. The experiment was performed according to the instructions of the TNF-α, IL-1β, IL-10 activity detection kit according to the instructions.

### 2.14. Statistical analysis

Data were analyzed by SPSS 18.0 and presented as the means ± standard deviation (SD). The Student’s t-test or the one-way ANOVA was used to evaluate the difference between groups. P values <0.05 were considered statistically significant.

## 3. Results

This study demonstrated that METTL14 was up-regulated in ox-LDL-incubated HUVECs. Knocking down METTL14 promoted viability and inhibited apoptosis of ox-LDL-incubated HUVECs. In addition, the p65 mRNA was a potential m6A target for METTL14. Overexpressing p65 reversed the effect of si-METTL14 on the viability and apoptosis of ox-LDL-incubated HUVECs.

### 3.1. METTL14 expression was upregulated in the ox-LDL-incubated HUVECs

We performed MTT assays and flow cytometry to explore the influence of different ox-LDL incubations (12 h or 24 h) on HUVEC viability and apoptosis. The viability of the HUVECs in the ox-LDL 12 h group was lower than that in the control group, and the ox-LDL 24 h group viability was lower than that of the ox-LDL 12 h group (Figure 1(a)). Furthermore, the apoptosis rate for the HUVECs in the ox-LDL 12 h group was higher than that in the control group, and the ox-LDL 24 h group had a higher apoptosis rate than the ox-LDL 12 h group (Figure 1(b,c)). ‘Writers’ (METTL3, METTL14, and WTAP) and ‘erasers’ (FTO, and ALKBH5) associated with the m^6^A process were evaluated by RT-qPCR. The results showed increased METTL3 and METTL14 expressions but reduced FTO expression in the ox-LDL treatment group compared to the control group. (Figure 1(d)). Flow cytometry analysis indicated that ox-LDL elevated the ROS activity of HUVECs (Figure 1(e)). ELISA results showed that ox-LDL promoted the release of TNF-α, IL-1β, and IL-10 (Figure 1(f)).

**Figure 1.** Cell viability and expression of key proteins associated with the N6-methyladenosine (m^6^A) process in ox-LDL incubated HUVECs. (a) cell viability of HUVECs detected by MTT after they had been incubated with ox-LDL for 12 h or 24 h. (b,c) apoptosis rates for HUVECs examined by flow cytometry with Annexin V-PE/7-AAD after they had been incubated with ox-LDL for 12 h or 24 h. (d) relative expressions of METTL3, METTL14, WTAP, FTO, and ALKBH5 in ox-LDL incubated HUVECs when detected by RT-qPCR assays. (e) Flow cytometry was used to detect the ROS activity. (f) ELISA was performed to detect the level of inflammatory factors including TNF-α, IL-1β, and IL-10. (N = 6). Asterisk (*) represents a statistical difference compared to the control group. Octothorp (#) represents a statistical difference compared to the ox-LDL 12 h group. ^*/#^*P* < 0.05, ^**/##^*P* < 0.001.g

### 3.2. Knocking down METTL14 promoted viability and inhibited apoptosis of ox-LDL-incubated HUVECs

The effects of METTL14 on the viability and apoptosis of ox-LDL-incubated HUVECs were explored by transfecting HUVECs with si-METTL14 to knock down its expression. Figure 2(a) shows that METTL14 expression in HUVECs decreased after transfection with si-METTL14 and the viability of ox-LDL-incubated HUVECs increased in the ox-LDL+si-METTL14 group compared to the ox-LDL+si-NC group (Figure 2(b)). The flow cytometry results revealed that the apoptosis rate was higher in the ox-LDL+si-NC group than in the control group, whereas it decreased in the ox-LDL+si-METTL14 group compared to the ox-LDL+si-NC group (Figure 2(c,d)). Western blotting showed increased expression of Bax and cleaved caspase-3 (c-cas3) in the ox-LDL+si-NC group compared to the control group, but a decreased antiapoptotic protein Bcl-2 expression in the ox-LDL+si-NC group compared to the control group (Figure 2(e,f)). Flow cytometry and ELISA results indicated that knockdown of METTL14 reversed the effect of ox-LDL on the ROS activity and release of TNF-α, IL-1β, and IL-10 in HUVECs (Figure 2(g,h)).

**Figure 2.** Influence of knocking down METTL14 on the apoptosis rates for ox-LDL incubated HUVECs. (a) relative expression of METTL14 in si-NC or si-METTL14 transfected HUVECs when detected by RT-qPCR. (b) viability of si-NC or si-METTL14 transfected cells examined by MTT assay after they had been incubated with ox-LDL. (c, d) apoptosis rate for si-NC or si-METTL14 transfected cells examined by flow cytometry with Annexin V-PE/7-AAD after they had been incubated with ox-LDL. (e, f) key proteins associated with the apoptosis process (bax, c-cas3, and bcl-2) in si-NC or si-METTL14 transfected cells when examined by Western blot after they had been incubated with ox-LDL. (g) Flow cytometry was used to detect the ROS activity. (h) ELISA was performed to detect the level of inflammatory factors including TNF-α, IL-1β, and IL-10. (N = 6). *P < 0.05, **P < 0.001.

### 3.3. The p65 mRNA was a potential m^6^A target for METTL14 in HUVECs

Potential m^6^A sites in mature p65 mRNA were first predicted and evaluated by SRAMP (Figure 3(a)). The m^6^A content in total RNA and relative m^6^A modification of p65 were evaluated. The results showed a decrease in total m^6^A levels in HUVECs after transfection with si-METTL14 compared to transfection with si-NC (Figure 3(b)). The Me-RIP assay also shows that m^6^A modification of p65 was also attenuated by METTL14 knockdown (Figure 3(c)). Further experiments revealed that the relative expression of p65 in HUVECs also decreased in the si-METTL14 group compared to that in the si-NC group (Figure 3(d)). Subsequently, we determined the mechanism by which METTL14 regulates the mRNA expression of p65. We determined the stability of p65 after METTL14 silencing. Interestingly, METTL14 knockdown significantly inhibited the stability of p65 (Figure 3(e)). The Western blotting results showed that nuclear and cytoplasmic p65 protein expression was both lower in the si-METTL14 group than in the si-NC group (Figure 3(f)).

**Figure 3.** Subunit p65 acts as a potential methylation target for METTL14 in HUVECs. (a) potential m^6^A sites in mature p65 mRNA were predicted and evaluated using SRAMP. (b, c) m^6^A content in total RNA or relative m^6^A level of the si-NC or si-METTL14 groups detected by RT-qPCR with the aid of a tool kit or an MeRIP assay. (d, e) relative expression of p65 at various time points (0, 3, 6, and 12 h) after actinomycin D application or 24 h after transfection with si-NC or si-METTL14 as detected by RT-qPCR. (f) Nuclear and cytoplasmic p65 expression was examined by Western blotting 24 h after transfection with si-NC or si-METTL14. (N = 4). *P < 0.05, **P < 0.001.

### 3.4. Overexpressing (OE) p65 could reverse the effect of si-METTL14 on the viability and apoptosis of ox-LDL-incubated HUVECs

Cells that overexpressed p65 were created by transfecting target cells with reconstructed pcDNA 3.1 vectors. These transfected cells were then used to evaluate the relationship between p65 and METTL14 and its effects on viability and apoptosis in the atherosclerosis cell model. The relative expression of nuclear and cytoplasmic p65 was significantly elevated in the OE-p65 group compared to that in the OE-NC group (Figure 4(a,b)). The MTT assays showed that viability in the ox-LDL+si-METTL14+ OE-NC group was higher than that in the ox-LDL+si-NC+OE-NC group. However, overexpression of p65 reversed the effect of si-METTL14, and led to a decrease in cell viability in the ox-LDL+si-METTL14+ OE-p65 group compared to the ox-LDL+si-METTL14+ OE-NC group (Figure 4(c)). The apoptosis rate was lower in the LDL+si-METTL14+ OE-NC group compared to the ox-LDL+si-NC+OE-NC group. The effect of si-METTL14 was reversed in the ox-LDL+si-METTL14+ OE-p65 group, and there was an increase in the apoptosis rate compared to the ox-LDL+si-METTL14+ OE-NC group (Figure 4(d,e)). Western blotting showed that the bax and c-cas3 expressions had decreased, while bcl-2 had increased in the ox-LDL+si-METTL14+ OE-NC group compared to the ox-LDL+si-NC+OE-NC group. In addition, the bax and c-cas3 levels increased, while that of bcl-2 decreased in the ox-LDL+si-METTL14+ OE-p65 group compared to the ox-LDL+si-METTL14+ OE-NC group (Figure 4(f,g)). Flow cytometry and LISA results indicated that overexpression of p65 reversed the effect of METTL14 on the ROS activity and release of TNF-α, IL-1β, and IL-10 in HUVECs (Figure 4(f,i)).

**Figure 4.** METTL14 interacted with p65, which influenced the apoptosis rates for ox-LDL-incubated HUVECs. (a) relative expression of p65 in HUVECs in the OE-NC and the OE-p65 groups when detected by RT-qPCR after transfection. (b) Western blot was used to evaluate the expression of p65. (c) viability of the HUVECs in the control, ox-LDL+si-NC+OE-NC, ox-LDL+si-METTL14+ OE-NC, and the ox-LDL+si-METTL14+ OE- p65 groups at various time points (0 h, 24 h, 48 h, and 72 h) when examined by MTT assays. (d, e) apoptosis rates for HUVECs in the control, ox-LDL+si-NC+OE-NC, ox-LDL+si-METTL14+ OE-NC, and the ox-LDL+si-METTL14+ OE- p65 groups when examined by flow cytometry with Annexin V-PE/7-AAD. (f, g) key proteins associated with the apoptosis process (bax, c-cas3, and bcl-2) in the control, ox-LDL+si-NC+OE-NC, ox-LDL+si-METTL14+ OE-NC, and ox-LDL+si-METTL14+ OE- p65 groups when detected by Western blotting. (h) Flow cytometry was used to detect the ROS activity. (i) ELISA was performed to detect the level of inflammatory factors including TNF-α, IL-1β, and IL-10. (N = 6). *P < 0.05, **P < 0.001.

### 3.5. Knocking down METTL14 could inhibit the formation of atherosclerosis in high-fat diet APOE^−/−^ mice

The relative expression of METTL14 in vascular tissue was first evaluated in the Ad-sh-METTL14, and the results showed a significant METTL14 decrease in the Ad-sh-METTL14 group compared to that in the Ad-sh-NC group (Figure 5(a)). The aorta specimens from the *APOE***^−/−^** mice showed that the Ad-sh-NC group had larger plaque areas than the control group after Oil Red O staining, whereas sh-METTL14 reversed this effect and the plaque area was smaller in the Ad-sh-METTL14 group compared to the Ad-sh-NC group (Figure 5(b)). A similar trend was also observed in the lesion areas of the aortic roots of the target mice. Specifically, the lesion areas were larger in the Ad-sh-NC group than in the control group after Oil Red O staining, whereas sh-METTL14 reversed this effect and the lesion areas were smaller in the Ad-sh-METTL14 group than in the Ad-sh-NC group (Figure 5(c)). Besides, in the Ad-sh-NC group, the protein expressions of p65 (Figure 5(d)), the cholesterol, triglyceride, and LDL-cholesterol levels were increased, and HDL-cholesterol levels (Figure 5(e)) were decreased compared with the control group, whereas sh-METTL14 reversed this effect. Furthermore, the immunofluorescence and TUNEL staining results showed CD31 was significantly decreased and apoptosis was significantly increased in the Ad-sh-NC group. While after sh-METTL14 transfection, these results were reversed (Figure 5(f)).

**Figure 5.** Effect of METTL14 on the formation of atherosclerosis in *APOE*^−/−^ mice. (a) relative expressions of METTL14 in the Ad-sh-NC or the Ad-sh-METTL14 groups when detected by RT-qPCR. (b) plaque areas of *APOE*^−/−^ mice aortas taken from the control, Ad-sh-NC, and the Ad-sh-METTL14 groups were examined and quantified using Oil Red O staining. (c) lesion areas (%) of the aortic roots in the control, Ad-sh-NC, and the Ad-sh-METTL14 groups were examined and quantified using Oil Red O staining. (N = 6). (d) protein expressions of p65 in control, Ad-sh-NC and the Ad-sh-METTL14 groups when detected by Western blot. (e) The levels of cholesterol, triglyceride, LDL-cholesterol and HDL-cholesterol in the control, Ad-sh-NC and the Ad-sh-METTL14 groups were detected by kits. (f) The CD31 levels and cell apoptosis in the the control, Ad-sh-NC and the Ad-sh-METTL14 groups were detected by immunofluorescence and TUNEL staining.*P < 0.05, **P < 0.001.

## 4. Discussion

Vascular endothelial cell damage plays an important role in the occurrence and development of AS [19,20]. When endothelial cells are in a normal physiological state, cell proliferation, and apoptosis are maintained in balance, which allows blood vessels to function normally [21]. When AS occurs, ox-LDL and other factors stimulate vascular endothelial cells, causing cells to undergo abnormal apoptosis, which damages the vascular tissue and ultimately leads to vascular dysfunction [22]. Therefore, this study established an ox-LDL-induced HUVEC model. The HUVECs induced by ox-LDL showed decreased proliferation and increased apoptosis, indicating that ox-LDL accelerated endothelial cell damage.

METTL3 and METTL14 are both methyltransferases that can transfer a methyl group to the adenosine bases [23]. An increasing number of studies have confirmed the critical role of METTL14 in m^6^A modification [24–26]. In addition, these METTL14 regulated m^6^A modifications participate in various biological processes, including RNA splicing, cell apoptosis, proliferation, and cell cycle arrest [27–29]. In this study, METTL14 expression was significantly upregulated in endothelial cells induced by ox-LDL. Furthermore, knocking out METTL14 significantly down-regulated the protein expressions of Bax and c-cas3, and up-regulated the Bcl-2 protein expression, which strongly suggested that METTL14 plays a vital role in the development of AS.

Subunit p65 plays a crucial role in the formation of nuclear factor κB, which is a well-known core transcription factor that regulates inflammation [30]. In the resting state without transcriptional activity, RelA (p65) and p50, which make up the NF-κB protein dimer, remain in the cytoplasm and bind to IκB. When stimulated by inflammatory factors, the upstream kinase IκB kinase (IKK) is activated, phosphorylates IκB (p-IκB), and degrades it due to ubiquitination [31]. NF-κB is one of the most critical inflammatory regulators of the pathological complications caused by AS and atherosclerotic thrombotic diseases [32,33]. NF-κB is involved in a variety of pathological processes during the formation of AS, such as foam cell production, endothelial cell apoptosis, inflammatory responses, and the pro-survival and pro-inflammatory state of blood vessels and blood cells [34,35]. Blockading NF-κB signaling has been reported to have a protective effect against AS [33,36,37]. NF-κB is the main transcription factor for the inflammatory response. It exists in the cytoplasm as homologous dimers or heterodimers during the resting state and remains inactive through interaction with inhibitors of κB (IκB) [38]. During the extracellular stimulation process caused by factors such as stress, cytokine bacteria, or viral antigens, NF-κB is dissociated from IκB and transported to the nucleus [39,40]. To further clarify the effect of METTL14, we analyzed data from SRAMP and revealed that p65 may be a downstream target of METTL14. METTL14-mediated m^6^A methylation influences p65 stability and its expression, and the results of this study show that overexpression of p65 can reverse the effect of METTL14 knockdown on ox-LDL-induced HUVEC injury.

We conducted in vivo experiments to further verify the effect of METTL14 knockdown on ox-LDL-induced HUVECs. The results showed that *APOE^−/−^* mice fed a high-fat diet had smaller plaques or lesions on their aortas after they had been injected with sh-METTL14.

## 5. Conclusion

Taken together, the present study clarifies the key role of METTL14 in the progression of human AS through the m^6^A-dependent modification of p65. This discovery and its impact on the development of AS will help further cardiovascular disease research and the development effective treatment strategies for AS.

## Supplementary Material

Supplemental Material
